The article "Changes of Tumor Markers in Patients with Lung Cancer after Immunotherapy and Their Link with Inflammation in the Body" was retracted in 2023. Reasons: signs of a paper mill; suspected computer-generated content; unreliable results or conclusions; concerns about the data.

# Changes of Tumor Markers in Patients with Lung Cancer after Immunotherapy and Their Link with Inflammation in the Body

**DOI:** 10.1155/2022/7781686

**Published:** 2022-07-19

**Authors:** LiWei Liu, YuanChun Cai, XiaoLan Tao, Jing Huang, Min Han

**Affiliations:** ^1^Department of Radiation Oncology, Maanshan People's Hospital, Maanshan City, Anhui Province 243000, China; ^2^Department of Oncology, Maanshan Shiqiye Hospital, Maanshan City, Anhui Province 243000, China

## Abstract

**Purpose:**

To figure out tumor markers changes in lung cancer (LC) patients after immunotherapy and their link with inflammation in the body.

**Methods:**

From May 2017 to January 2021, taking 97 LC patients with elevated Programmed Cell Death Protein 1 and Programmed Cell Death Protein-ligand 1 was as the research objects. They were all given immunotherapy and assigned into the remission and the nonremission groups on the grounds of the tumor remission after 6 months of treatment, after comparison of tumor markers [carcinoembryonic antigen (CEA), squamous cell carcinoma-associated antigen (SCC-Ag), cytokeratin 19 fragment (CYFRA12-1), and neuron-specific enolase (NSE)] and inflammation indicators [interleukin-10 (IL-10), interleukin (IL-6), and tumor necrosis factor-*α* (TNF-*α*)] in the two.

**Results:**

Tumor markers, IL-10, IL-6, and TNF-*α* in the remission after treatment were reduced vs. the nonremission (*P* < 0.05); SCC-Ag was positively linked with IL-10, IL-6, and TNF-*α* in the patients after treatment (*P* < 0.05); the AUC of the combined detection to assess the efficacy of LC immunotherapy was greater vs. the individual detection of indicators (*P* < 0.05).

**Conclusion:**

Tumor markers and the inflammation state of the body in LC patients are memorably reduced after immunotherapy, and a correlation is presented between the two, which manifests evaluating value of the efficacy of immunotherapy.

## 1. Introduction

Lung cancer (LC) is a malignant tumor with surprising morbidity and mortality in China, and its presence is elevated year by year. It is currently believed that besides factors like genetics and social influence, immune escape mechanisms are also crucial in LC's presence and advancement [1]. Relevant studies have pointed out when the patient's immunity is reduced or suppressed, the tumor progression rate is memorably accelerated [2]. Hence, immunotherapy, as a novel kind of adjuvant cure for cancer patients, has been gradually applied to the clinic. Recently, the immune evasion induced via the combination of Programmed Cell Death Protein 1 (PD-1) and Programmed Cell Death Protein-ligand 1 (PD-L1) has become an impactive target for tumor cure, bringing a new direction for advanced LC therapy [3]. Immunotherapy is available to motivate the recovery of the body's immune function and eliminate the concealed micrometastasis of tumor cells that cannot be discovered and eradicated via conventional methods, thereby achieving a better therapeutic effect. A relevant report has clarified immunotherapy does not lead to fatal side effects similar with chemotherapy and radiotherapy to the body [4]. However, the link of the changes of serum tumor markers and the inflammatory state in LC patients after immunotherapy is still uncertain. Hence, the study was for figuring out tumor marker changes in LC patients after immunotherapy and their link with inflammation in the body, offering reference for clinical cure of the disease.

The article "Changes of Tumor Markers in Patients with Lung Cancer after Immunotherapy and Their Link with Inflammation in the Body" was retracted in 2023. Reasons: signs of a paper mill; suspected computer-generated content; unreliable results or conclusions; concerns about the data.

## 2. Materials and Methods

### 2.1. Clinical Data

From May 2017 to January 2021, taking 97 LC patients with elevated PD-1 and PD-L1 was as the research objects. The patients were all given immunotherapy and assigned into remission (*n* = 61) and nonremission (*n* = 36) groups on the grounds of the tumor remission after 6 months of treatment, and no clear difference was presented in general data between the two (Table 1, *P* > 0.05). Written informed consent was obtained from all participants, and the present study was approved by the Institutional Review Board of Maanshan People's Hospital.

### 2.2. Inclusion Criteria

Inclusion criteria are as follows: ① complying with the diagnostic criteria for LC in the *Guidelines for the Diagnosis and Treatment of Primary Lung Cancer in China (2015 Edition)* [5]; ② patients undergoing immunotherapy; ③ age ≥ 18 years; ④ one with elevated PD-1 and PD-L1.

### 2.3. Exclusion Criteria

Exclusion criteria are as follows: ① severe heart and liver dysfunction; ② patients with cardiovascular and cerebrovascular diseases; ③ those having a history of immunotherapy; ④ patients with other malignant diseases; ⑤ those with contraindications to immunotherapy; ⑥ expected survival time of less than 6 months.

### 2.4. Methods

#### 2.4.1. Immunotherapy Methods

All were given nivolumab injection (Bristol-Myers Squibb Holdings Pharma, Ltd., batch number: registration number S20180015, specification: 100 mg/10 ml), with 3 mg/kg dose, intravenous drip for 60 min, once/2 w treatment frequency, and a total of 6 cycles of treatment.

#### 2.4.2. Efficacy Evaluation Criteria

Referring to *Solid Tumor Curative Effect Evaluation Standard (RECIST) 1.1* [6], the therapeutic effect was evaluated and assigned into complete remission, partial remission, stable disease, and progress. On the grounds of the effect, assignation of patients was into remission (complete remission, partial remission) and nonremission groups.

The article "Changes of Tumor Markers in Patients with Lung Cancer after Immunotherapy and Their Link with Inflammation in the Body" was retracted in 2023. Reasons: signs of a paper mill; suspected computer-generated content; unreliable results or conclusions; concerns about the data.

#### 2.4.3. Detection of Tumor Markers

Application of the ELECYS automatic electrochemiluminescence immunoassay detector from Roche (Germany) was for detecting the carcinoembryonic antigen (CEA), squamous cell carcinoma antigen (SCC-Ag), cytokeratin 19 fragment antigen21-1 (CYFRA12-1), and neuron-specific enolase (NSE) in patients before and after treatment.

### 2.5. Observation Indicators

(1) Comparison of tumor markers and inflammation indicators of the two groups and analysis the link between the two were conducted; (2) analysis of the evaluation value of tumor markers and inflammatory indexes for the efficacy of LC immunotherapy and their link with tumor remission.

### 2.6. Statistical Processing

Application of SPSS22.0 software was to process the data; manifestation of count data was in %, and comparison of the difference of groups was via *χ*^2^ test. Manifestation of measurement data was as ($\bar{x}\pm s$) after normal test, and comparison of the difference of groups was via *t* test. Receiver-operator characteristic (ROC) curve was employed for analysis of the evaluation value of tumor markers and inflammatory indexes on the efficacy of LC immunotherapy, with the Pearson test for analysis of the link of tumor markers and inflammatory indexes in patients after treatment, and multivariate logistic regression for analysis of the connection of tumor markers and inflammatory indexes and the efficacy of LC immunotherapy. *P* < 0.05 emphasized obvious statistical meaning.

## 3. Results

### 3.1. Comparison of Tumor Markers before and after Treatment in the Remission and the Nonremission

Tumor markers in the remission after treatment were reduced vs. the nonremission (*P* < 0.05), as manifested in Figure 1.

### 3.2. Comparison of Inflammation Indexes

After treatment, IL-10, IL-6, and TNF-*α* in the remission were declined vs. the nonremission (*P* < 0.05), as manifested in Figure 2.

### 3.3. The Link Analysis of Tumor Markers and Inflammatory Indexes in Patients after Treatment

In the patients after treatment, the SCC-Ag was positively linked with IL-10, IL-6, and TNF-*α* (*P* < 0.05), as clarified in Figure 3.

Neural machine translation: the proposal of neural machine translation provides a faster and more accurate translation method for machine translation. However, most language pairs have only a few hundred to thousands of parallel sentences. The lack of data is a serious problem for training a suitable machine translation system. Because both neural machine translation (NMT) and statistical machine translation (SMT) are highly dependent on data, the data dependency of both NMT and SMT is high.

The article "Changes of Tumor Markers in Patients with Lung Cancer after Immunotherapy and Their Link with Inflammation in the Body" was retracted in 2023. Reasons: signs of a paper mill; suspected computer-generated content; unreliable results or conclusions; concerns about the data.

### 3.4. Analysis of the Evaluation Value of Tumor Markers and Inflammatory Indexes on the Efficacy of LC Immunotherapy

The AUC of combined detection to evaluate the efficacy of LC immunotherapy was greater vs. individual detection of indexes (Table 2 and Figure 4, *P* < 0.05). This indication was approved based on the phase III efficacy confirmatory clinical trial checkmate-816. Checkmate-816 is a randomized, open label phase III clinical study conducted in multiple centers to evaluate the efficacy of drug o combined with chemotherapy in the neoadjuvant stage of resectable non-small-cell lung cancer compared with chemotherapy alone, regardless of the tumor PD-L1 expression level. The results of this study showed that compared with chemotherapy alone (chemotherapy group), drug o combined with chemotherapy (immunotherapy group) reduced the risk of disease progression, recurrence or death by 37% (hr = 0.63). In addition, the median event-free survival (EFS) was 31.6 months in the immunochemotherapy group and only 20.8 months in the chemotherapy group. Among the pathological remission indexes, the complete pathological remission (PCR) in the combined treatment group was 24%, while that in the chemotherapy group was only 2.2% (Table 2). In terms of safety, the safety of drug o combined with chemotherapy group was consistent with previous studies on non-small-cell lung cancer. As the first neoadjuvant phase III clinical trial of lung cancer immunization, checkmate-816 confirmed that neoadjuvant immunization combined with chemotherapy can bring clinical benefits to patients with resectable non-small-cell lung cancer.

### 3.5. Logistic Regression Analysis of Tumor Markers and Inflammation Indexes and the Efficacy of LC Immunotherapy

CEA ≥ 53.74 ng/ml, SCC − Ag ≥ 1.49 ng/ml, IL − 10 ≥ 16.95 pg/ml, and IL − 6 ≥ 0.76 pg/ml were risk factors impacting the efficacy of LC immunotherapy (Table 3, *P* < 0.05).

## 4. Discussion

The present drug treatment of LC majorly consists of immunotherapy, chemotherapy, and targeted therapy. However, more patients are intolerant of the adverse reactions of chemotherapy drugs, greatly declining the antitumor impact and probably affecting the quality of life of patients [7, 8]. In the context of precision medicine, targeted and immunotherapy have been gradually employed to the clinic, giving patients the chance of long-term survival. The principle of immunotherapy is majorly that the surface of T cells represses their activation and participate in the signal pathway of immune response. In the tumor microenvironment, the function of T cells is refrained, and it cannot kill tumor cells [9]. The interaction of PD-1 and PD-L1 is the crux to tumor immune escape, repressing T cell activation and proliferation, thereby mediating negative immune modulation. Implicated reports point out immunotherapy is available to be applied as a brand-new method for LC cure [10, 11]. During LC advancement, tumor cells via expressing PD-1 and PD-L1 transform the tumor microenvironment into immunosuppression, ultimately inducing tumor cells evading the surveillance of the immune system and motivating tumor progression [12]. This study discovered tumor markers in the remission after treatment was reduced vs. the nonremission, clarifying that effective immunotherapy is available to repress tumor growth, which is mainly linked with immunotherapy reversing T lymphocyte depletion and motivating the recovery of antitumor immune function.

The article "Changes of Tumor Markers in Patients with Lung Cancer after Immunotherapy and Their Link with Inflammation in the Body" was retracted in 2023. Reasons: signs of a paper mill; suspected computer-generated content; unreliable results or conclusions; concerns about the data.

Linked reports point out LC patients are generally in a state of elevated inflammation, which is majorly induced via the patient's psychological stress and the translation of inflammatory factors by tumor cells. Elevated inflammation is available to further constitute the microenvironment for tumor growth, resulting in patients with nerve axis function disorders and other phenomena [13, 14]. TNF-*α* and others are specific factors for LC patients, which can reflect inflammation in patients [15]. Immunotherapy is available to strengthen humoral immunity, augment the body's immune response, activating T cells to attack their own normal tissues, and stimulate autoimmune responses [16, 17] [18]. The results of this study manifested the AUC of combined detection to evaluate the efficacy of LC immunotherapy was greater vs. individual indicators, manifesting that the combined detection of various indicators has an evaluation value for the efficacy of LC immunotherapy, suggesting that it might be applied in the clinical evaluation of immunotherapy for LC patients.

Tumor markers refer to substances characteristically present in malignant tumor cells, or abnormally produced via malignant tumor cells or the host's response to tumor stimulation. They majorly exist in tumor cells or in the patient's body fluid, which can reflect the existence and growth of tumors [19, 20]. Inflammation also takes on an essential character in the occurrence and development of tumors. The stimulation of chronic inflammation can lead to tumors to release many factors directly motivating their own growth, which constitutes an inflammatory microenvironment conducive to tumors' presence and advancement. The inflammatory response also impacts the host's immune response to tumors [21, 22]. Related reports point out inflammation has a tumor-promoting impact [23]. Tumor development induced via inflammatory response may show up in the early or late stage of the tumor and can lead to the activation of dormant cancer cells [24, 25]. Therefore, the author believed tumor markers in LC patients might be linked with inflammatory factors. This study discovered SCC-Ag was positively linked with IL-10, IL-6, and TNF-*α* after treatment, indicating that inflammation in patients was implicated in tumor markers, which might be associated with tumors' presence and advancement. This study clarified CEA ≥ 53.74 ng/ml, SCC − Ag ≥ 1.49 ng/ml, IL − 10 ≥ 16.95 pg/ml, and IL − 6 ≥ 0.76 pg/ml were risk factors impacting the efficacy of LC immunotherapy, indicating that elevated tumor markers and inflammation could affect the efficacy of immunotherapy in patients. The reason is still unknown, so further analysis is required in the later stage.

The article "Changes of Tumor Markers in Patients with Lung Cancer after Immunotherapy and Their Link with Inflammation in the Body" was retracted in 2023. Reasons: signs of a paper mill; suspected computer-generated content; unreliable results or conclusions; concerns about the data.

In short, tumor markers and the inflammation state of the body in LC patients are memorably reduced after immunotherapy, and a correlation is presented between the two, which manifests evaluating value of the efficacy of immunotherapy.

## Figures and Tables

**Figure 1:** Comparison of tumor markers vs. the remission after treatment, ^∗^*P* < 0.05.

**Figure 2:** Comparison of inflammation indexes before and after treatment in the remission and the nonremission (pg/ml) vs. the remission after treatment, ^∗^*P* < 0.05.

**Figure 3:** Correlation analysis of tumor markers and inflammation indexes in patients after treatment.

**Figure 4:** ROC curve analysis of combined detection of tumor markers and inflammatory indexes to evaluate the efficacy of LC immunotherapy.

**Table 1:** Comparison of general data between the remission and the nonremission.

Groups	The remission (*n* = 61)	The nonremission (*n* = 36)	*χ* ^2^/*t*	*P*
Gender male (cases)	37	21	0.013	0.910
Age	59.37 ± 6.18	60.42 ± 6.59	0.789	0.432
BMI (kg/m^2^)	21.53 ± 2.51	21.89 ± 2.68	0.665	0.507
Pathological type			0.122	0.941
Squamous carcinoma	28	16		
Adenocarcinoma	20	13		
Large cell carcinoma	13	7		
Staging			0.077	0.781
Stage IIIB	39	22		
Stage IV	22	14		
Family history of LC	6	2	0.548	0.459
Smoking history	31	15	0.761	0.383
Drinking history	24	11	0.758	0.384

**Table 2:** Analysis of the evaluation value of tumor markers and inflammatory indexes for the efficacy of LC immunotherapy.

Indexes	Cut-off point	AUC	SE	95% CI
CEA	53.74 ng/ml	0.662	0.060	0.545~0.779
SCC-Ag	1.49 ng/ml	0.707	0.055	0.599~0.815
CYFRA12-1	7.25 ng/ml	0.798	0.045	0.709~0.886
NSE	61.03 ng/ml	0.823	0.041	0.743~0.903
IL-6	16.95 pg/ml	0.683	0.054	0.576~0.789
IL-10	0.76 pg/ml	0.790	0.045	0.701~0.878
TNF-*α*	19.47 pg/ml	0.738	0.050	0.640~0.836
Combined detection		0.975	0.012	0.951~0.999

**Table 3:** Logistic regression analysis of tumor markers and inflammation indexes and the efficacy of LC immunotherapy.

Indexes	*β*	SE	Wald *χ*^2^	OR	95% CI	*P*
CEA	0.324	0.146	4.925	1.383	1.039~1.841	0.027
SCC-Ag	1.451	0.523	7.697	4.267	1.531~11.895	0.006
CYFRA12-1	0.645	0.377	2.927	1.906	0.910~3.991	0.088
NSE	0.348	0.221	2.480	1.416	0.918~2.184	0.116
IL-6	0.521	0.096	29.453	1.684	1.395~2.032	<0.001
IL-10	0.630	0.225	7.840	1.878	1.208~2.918	0.005
TNF-*α*	1.465	0.965	2.305	4.328	0.653~28.686	0.130
Constant term	-1.898	0.267	50.532	0.150	0.089~0.253	<0.001

Assignment: clinical efficacy (invalid was 1, effective was 0); CEA (≥53.74 ng/ml, 1; <53.74 ng/ml, 0); SCC-Ag (≥1.49 ng/ml, 1; <1.49 ng/ml, 0); CYFRA12-1 (≥7.25 ng/ml, 1; <7.25 ng/ml, 0); NSE (≥61.03 ng/ml, 1; <61.03 ng/ml, 0); IL-10 (≥16.95 pg/ml, 1; <16.95 pg/ml, 0); IL-6 (≥0.76 pg/ml, 1; <0.76 pg/ml, 0); TNF-*α* (≥19.47 pg/ml, 1; <19.47 pg/ml, 0).

The article "Changes of Tumor Markers in Patients with Lung Cancer after Immunotherapy and Their Link with Inflammation in the Body" was retracted in 2023. Reasons: signs of a paper mill; suspected computer-generated content; unreliable results or conclusions; concerns about the data.

## Data Availability

The experimental data used to support the findings of this study are available from the corresponding author upon request.
